The article "Neuron tau-targeting biomimetic nanoparticles for curcumin delivery to delay progression of Alzheimer’s disease" was retracted in 2023. Reasons: manipulated images; errors in the images; original data or images not available; unreliable data.

# Neuron tau-targeting biomimetic nanoparticles for curcumin delivery to delay progression of Alzheimer’s disease

**DOI:** 10.1186/s12951-020-00626-1

**Published:** 2020-05-13

**Authors:** Chunhong Gao, Xiaoyang Chu, Wei Gong, Jinpeng Zheng, Xiangyang Xie, Yuli Wang, Meiyan Yang, Zhiping Li, Chunsheng Gao, Yang Yang

**Affiliations:** 1 State Key Laboratory of Toxicology and Medical Countermeasures, Beijing Institute of Pharmacology and Toxicology, Beijing, 100850 China; 2 The Fifth Medical Center of Chinese, PLA General Hospital, Beijing, 100071 China; 3 General Hospital of Central Theater of the PLA, Wuhan, 430070 China

**Keywords:** Neuronal p-tau-targeting, Blood–brain barrier, Biomimetic nanosystems, Alzheimer’s disease, CUR

## Abstract

**Background:**

Although many therapeutic strategies for Alzheimer’s disease (AD) have been explored, these strategies are seldom used in the clinic. Therefore, AD therapeutic research is still urgently needed. One major challenge in the field of nanotherapeutics is to increase the selective delivery of drugs to a targeted location. Herein, we devised and tested a strategy for delivery of nanoparticles to neurons to inhibit tau aggregation by directly targeting p-tau.

**Results:**

Curcumin (CUR) is loaded onto red blood cell (RBC) membrane-coated PLGA particles bearing T807 molecules attached to the RBC membrane surface (T807/RPCNP). With the advantage of the suitable physicochemical properties of the PLGA nanoparticles and the unique biological functions of the RBC membrane, the RPCNP are stabilized and promote sustained CUR release, which provided improved biocompatibility and resulted in long-term presence in the circulation. Under the synergistic effects of T807, T807/RPCNP can not only effectively penetrate the blood–brain barrier (BBB), but they also possess high binding affinity to hyperphosphorylated tau in nerve cells where they inhibit multiple key pathways in tau-associated AD pathogenesis. When CUR was encapsulated, our data also demonstrated that CUR-loaded T807/RPCNP NPs can relieve AD symptoms by reducing p-tau levels and suppressing neuronal-like cells death both in vitro and in vivo. The memory impairment observed in an AD mouse model is significantly improved following systemic administration of CUR-loaded T807/RPCNP NPs.

**Conclusion:**

Intravenous neuronal tau-targeted T807-modified novel biomimetic nanosystems are a promising clinical candidate for the treatment of AD.

## Background

The complex multifactorial nature of polygenic Alzheimer’s disease (AD) presents challenges for drug development. Although numerous studies suggest removing amyloid-β (Aβ) deposits is “a promising therapeutic strategy”, almost all the Aβ-targeting drug candidates have failed in clinical trials [1–3]. These failures cast doubt on the amyloid cascade hypothesis. Recent studies have shown that the tau pathology can take place independently of Aβ and demonstrates a stronger correlation with clinical development of AD symptoms, which might be a potential therapeutic target [4]. Tau is a microtubule-associated protein found in the central nervous system (CNS) and peripheral nervous system, where it is primarily located in the axons of healthy neurons. Localization of tau in the neuron is largely dependent on post-translational modifications, most notably phosphorylation. Phosphorylated tau is generally sequestered in the soma of neurons, with small traces founded in the nucleus [5]. Similar to other microtubule-associated proteins, tau preserves microtubule stability and monitors intracellular trafficking [6]. However, in AD, the normal function of tau is interrupted, and a large amount of phosphorylated tau accumulates. Phosphorylation of tau decreases its affinity for microtubules, thereby decreasing overall tubulin assembly, which leads to the development of intraneuronal neurofibrillary tangles (NFTs) [7]. NFTs are formed from phosphorylated tau aggregates and remain intracellular until the neuron dies [8]. Furthermore, tau function is impaired, which also increases mitochondrial function burden, leading to mitochondrial dysfunction and reactive oxygen species (ROS) release [9]. Therefore, therapeutic agents that target tau pathology, repair abnormal tau and restrain a series of reactions caused by abnormal tau could be of great value for AD treatment [10]. In recent years, numerous tau-relevant and druggable mechanistic targets have been identified within tau pathology, but efforts to address this source of pathology have not been translated into clinically effective therapies [11]. Efficacy can be hindered by both the failure to attain adequate intraneuronal drug concentrations and the occurrence of off-target effects on extraneuronal machinery [12].

The article "Neuron tau-targeting biomimetic nanoparticles for curcumin delivery to delay progression of Alzheimer’s disease" was retracted in 2023. Reasons: manipulated images; errors in the images; original data or images not available; unreliable data.

Nowadays, nanotechnology represents a promising approach for the delivery of therapeutic agents to the CNS [13]. The sustained and precise drug targeting ability of nanotechnology could compensate for the defects of insufficient drug concentrations in the CNS. However, an ideal nanoparticle used in CNS drug delivery should efficiently cross the blood–brain barrier (BBB) and be specific enough to reach the targeted sites; the ideal nanoparticle would also have suitable physiochemical features, good biocompatibility and efficient scale-up for production. To date, several tau-targeted nanomaterials have been used to deliver drugs for the treatment of AD: Behafarid et al. prepared folic acid-functionalized gold nanoparticles (FA-AuNPs) and Gold-Fe_3_O_4_ core–shell nanoparticles (AuFeNPs), which exhibited binding affinity for both tubulin and tau [14]; Shweta et al. [15] found that protein-capped metal nanoparticles could inhibit tau aggregation in Alzheimer’s disease. However, problems with some of these inorganic nanomaterials still exist, such as difficult biodegradation in vivo and intolerable adverse side effects. Several organic nanomaterials, such as PLGA, have been approved as promising pharmaceutical delivery platforms due to their excellent biocompatibility, low cytotoxicity and biodegradability [16]. Several types of drug-loaded PLGA nanoparticles have been reported to reverse cognitive deficits in an AD transgenic mouse model [17]. However, PLGA-based nanotherapies still suffer from low BBB penetration ability and unstable circulation in the blood stream [18].

T807 (AV-1451), a novel tau positron emission tomography imaging agent for Alzheimer’s disease, exhibits strong binding to phosphorylation tau positive human brain sections [19]. Due to its lower molecular weight and suitable logP (1.5), it can effectively cross the blood–brain barrier (BBB) and it possesses cell permeability, and since it is safe in vivo, it is now widely used in the clinic to detect tau pathology [20]. This highly selective and p-tau-specific tracer also has a relatively high permeability for neurons, which are the main areas of tau aggregation [21]. All these beneficial features provide a chance to use T807 as a target ligand and AD therapeutic agent for delivery into the brain. Red blood cell membranes, termed RBCm, are extracted from red blood cells. They are thus readily available and abundant in the body and are convenient for scaling up and cost-effective preparation. The coating of the surface of nanoparticles (RPCNP) with intact RBCm endows RBCNPs with both the physicochemical properties of synthetic materials and the complex biological functions of endogenous materials [22]. Its low immunogenicity and long half-life in the circulation in vivo make it popular for drug delivery [23].

Multi-target drug candidates, such as curcumin (CUR), have been developed for the polygenic features of AD. CUR is a natural product of the curcuma longa plant that has been used in cooking and herbal medicine for centuries and that has been demonstrated to be a safe and effective agent in the central nervous system [24]. Recent data in the literature showed that CUR may also induce positive and very encouraging effects on neurogenesis and neuronal differentiation pathways. For example, CUR exerts neuroprotective effects by activating brain-derived neurotrophic factor/TrkB-dependent MAK and PI-3K cascades in rodent cortical neurons [25], and it has exhibited many promising abilities for incurable neurodegenerative and neuropsychiatric disorders that exact a huge toll on society [26]. Currently, CUR is being tested in phase II clinical trials as a tau-targeting agent [27, 28]. Therefore, it is a very promising therapeutic agent for AD. However, CUR is almost insoluble in water, has a very short half-life and low bioavailability, and it is photodegradable and chemically unstable at neutral physiological pH [29]. Considering the clinical therapeutic potential in that CUR could restrain tau hyperphosphorylation and decrease hyperphosphorylated tau aggregation [30], combination nanotechnology that can improve its bioavailability in the brain represents a promising strategy for AD treatment and is highly desired.

The article "Neuron tau-targeting biomimetic nanoparticles for curcumin delivery to delay progression of Alzheimer’s disease" was retracted in 2023. Reasons: manipulated images; errors in the images; original data or images not available; unreliable data.

Here, we report the design and synthesis of functionalized RBCm-coated nanoparticles with DSPE-PEG_3400_-T807 (T807) that can effectively cross the BBB and precisely target tau within neuronal cells. Conjugation of a T807 group to various small molecules or even to a drug delivery system can facilitate their strong brain-targeting ability [31]. We used a lipid-insertion method to combine the T807 ligand and RBCm-coated nanoparticles [32]. T807 combined with RBCm could effectively increase the BBB permeation of CUR and its circulation in the blood, which further enhanced the sustained exposure of the brain and the lesion sites to the drugs. A working sketch of these biomimetic, engineered delivery nanosystems (T807/RPCNP) is shown in Fig. 1. The results show that, with T807, this delivery nanosystem efficiently crossed the BBB, after which the RPCNP accumulated primarily in neurons. By loading CUR, the biomimetic nanosystems effectively prevent the pathogenic process of AD. In this article, the physicochemical and biological characterization of the T807/RPCNP was performed both in vitro and in vivo, and the underlying mechanism of the therapeutic effect was further investigated in vitro. Moreover, the in vivo therapeutic evaluations of CUR-loaded T807/RPCNP were also explored in an OA-induced AD mouse model.

**Fig. 1:** **a** Schematic interpretation of T807/RPCNP-CUR in vivo. According to the precise targeting of T807, the novel biomimetic engineered delivery nanosystems accumulate in neurons after crossing the BBB. **b** The preparation of T807/RPCNP-CUR. First, the RBCm was derived from RBCs and bare NPs were prepared using an emulsification ultrasonication method. Next, the resulting RBC membranes were coated onto the surface of bare NPs through mechanical extrusion to form RPCNP-CUR. Finally, DSPE-PEG_3400_-T807 was inserted into the outer monolayer of RBCm to form T807/RPCNP-CUR NPs

The article "Neuron tau-targeting biomimetic nanoparticles for curcumin delivery to delay progression of Alzheimer’s disease" was retracted in 2023. Reasons: manipulated images; errors in the images; original data or images not available; unreliable data.

## Materials and methods

### Materials

Amino-T807 and 1, 2-distearoyl-sn-glycero-3-phosphoethanolamine-*N*-hydroxy succinimide (NHS) (DSPE-PEG3400-NHS) was provided by Xi’an ruixi Biological Technology Co., Ltd (Xi’an, China). PLGA (Mw: 56 kDa) with a lactic/glycolic acid ratio of 75/25 was obtained from Jinan Daigang Biological Technology Co., Ltd (Shandong, China). CUR was purchased from Yuanye Biotechnology Co, Ltd (Shanghai, China). 1, 1′-Dioctadecyl-3, 3, 3′, 3′-tetramethylindotrica-rbocyanine iodide (DIR) and coumarin (COU 6) were purchased from Beijing Perenley Biotechnology Co., Ltd (Beijing, China). All chemicals were of reagent grade and were obtained from Sigma-Aldrich, unless otherwise stated.

### Synthesis of DSPE-PEG3400-T807

DSPE-PEG_3400_-T807 was synthesized through an NHS-amino coupling reaction. Briefly, the amino-T807 was dissolved in chloroform and added to DSPE-PEG_3400_-NHS at an amino-T807 to lipid molar ratio of 1.5:1. The mixture was gently stirred overnight at room temperature in the dark. The resultant supernatant was dialyzed against distilled water for 48 h. The purified dialysate was lyophilized and stored at − 20 °C.

### RBCm derivation

RBCm of ICR mice were collected according to a previously reported method [33]. In a nutshell, fresh whole blood was collected from female ICR mice (20 ± 2 g) and then centrifuged at 3000×*g* for 10 min at 4 °C to separate the plasma and the buffy coat. The resultant RBCm were treated with a hypotonic solution, and finally, the harvested RBCm were dispersed by ultrasonication (output power 200 W, time 3 min). The obtained vesicles were subsequently extruded serially through 400, and 200 nm polycarbonate porous membranes, and then stored in PBS at 4 °C until use.

### Preparation of PLGA nanoparticles

PLGA nanoparticles (NPs) were prepared using the O/W emulsion method. Briefly, 15 mg of PLGA and 1.25 mg of CUR or hydrophobic probe (DIR or COU 6) were added to 2 mL of an acetone mixture. When completely dissolved, the mixture was poured into 4 mL of pH 7.4 PBS buffer solution for 1 h. Then, the mixture was emulsified by ultrasonication (output power 300 W, time 5 min), and finally, the acetone solvent was removed by rotating the evaporator to form CUR-loaded PLGA NPs or hydrophobic probe-labelled PLGA NPs.

The CUR encapsulation efficiency (EE) and drug loading capacity (DL) of the formulation was determined by minicolumn centrifugation using HPLC to quantify the CUR in the NPs (EE% = (W_total CUR_ − W_free__CUR_)/W_total drug_ × 100%; EE: 90.23 ± 1.25%. DL% = (W_total drug_ − W_free drug_)/W_total drug_ and carriers × 100%; DL: 4.87 ± 1.04%).

The article "Neuron tau-targeting biomimetic nanoparticles for curcumin delivery to delay progression of Alzheimer’s disease" was retracted in 2023. Reasons: manipulated images; errors in the images; original data or images not available; unreliable data.

### Preparation of T807-RPCNP nanoparticles

Biomimetic nanoparticles included plain RBCm-PLGA nanoparticles (RPCNP NPs, without targeting ligand) and RPCNP with the DSPE-PEG_3400_-T807 modification (T807-RPCNPs). For RPCNP, RBCm coating was completed by fusing RBCm vesicles with NPs via sonication in a bath sonicator (SCIENTZ-IID, Zhengjiang, China) with 100 W power (working model: work 3 s and stop 10 s), and then extruded 10 times through a 200 nm polycarbonate porous membrane using a mini extruder (Avanti Polar Lipids, USA), T807-RPCNPs were formed by the post-insertion method. Briefly, DSPE-PEG_3400_-T807 (23 mg) and RPCNPs (25 mg) were mixed in 10 mL of pH 7.4 PBS solution, which was followed by sonication. The brown suspension was filtered in a syringe filter with a 0.45 µm pore size. To remove free PEG_3400_-T807, we purified the T807-RPCNPs thoroughly by dialysis using a dialysis bag with a 10 kDa molecular weight cut off (Thermo, Rockford, IL, USA) for 24 h.

### Characterization of biomimetic nanoparticles

The mean diameter, particle distribution and zeta potential of these biomimetic nanoparticles were measured by dynamic light scattering (DLS) (Litesizer 500, Anton Parr, Austria). The morphology of these biomimetic nanoparticles was characterized using transmission electron microscopy (TEM) (HITACHI, H-7650, Japan). The stability of these biomimetic nanoparticles in whole mouse serum was evaluated using a Turbiscan Lab^®^ Expert (Formulaction, L’Union, France). The stability analysis was performed with the instrument software as a variation of Delta Transmission (ΔT) and Backscattering (ΔBS) profiles.

Sodium dodecyl sulfate-polyacrylamide gel electrophoresis (SDS-PAGE) was used to analyze the proteins. Proteins in T807-RPCNPs, RBC lysate and RBCm were prepared in SDS sample buffer (Invitrogen, USA) and measured using a Bicinchoninic (BCA) assay kit (Pierce, China). The structural information of CD47 was characterized by a J-810 circular dichroism (CD) spectrometer (JASCO, Japan). Detailed immunoblotting procedures have been previously described [34].

### In vitro release profile

In vitro drug release studies were performed with some modifications since CUR degrades in alkaline solutions [35]. Briefly, CUR, freeze-dried CUR-RPCNPs and CUR-PCNPs (∼ 1 mg CUR in each) containing equal amounts of CUR were each suspended in 120 mL phosphate-buffered saline (0.1 M, pH 7.4); the CUR solution was divided into eight parts, and each part contained three samples, which were then placed in a shaking incubator (180 cycles/min) at 37 °C. Sampling was performed at 30 min, 1 h, 2 h, 4 h, 6 h, 8 h, 12 h, and 24 h. After centrifugation at 2500 rpm for 10 min, the sediments were collected, diluted, and analyzed by HPLC. Experiments were performed in triplicate.

The article "Neuron tau-targeting biomimetic nanoparticles for curcumin delivery to delay progression of Alzheimer’s disease" was retracted in 2023. Reasons: manipulated images; errors in the images; original data or images not available; unreliable data.

### Cell culture

In accordance with a previous report, primary brain capillary endothelial cells (RBMVECs) were purchased from iCell Bioscience Inc (Shanghai, China). Astrocytes (As) were isolated from 3-day Sprague–Dawley (SD) rats and maintained in Astrocyte Basal Medium-2 (iCell Bioscience Inc, Shanghai, China). HT22 cells (a neuronal-like cell line) were purchased from the Cell Resource Centre of IBMS (Beijing, China) and were maintained in culture medium consisting of Dulbecco’s Modified Eagle’s Medium (DMEM) supplemented with 10% FBS, 100 IU/mL penicillin, and 100 mg/mL streptomycin. These cells were maintained in a 37 °C humidified incubator in an atmosphere of 5% CO_2_. All antibodies were purchased from Abcam Co, Ltd (England).

### Cytotoxicity of biomimetic nanoparticles

HT22 cells were seeded onto 96-well plates (5 × 10^3^ cells/well) for 24 h and then treated with or without OA (40 nM/L). After incubation for 12 h, the cells were treated with different concentrations of CUR-loaded biomimetic nanoparticles (5 µg/mL CUR, with OA) and bare biomimetic nanoparticles (without OA) and incubated for another 12 h. At the end of the incubation, cell viability was evaluated by methyl thiazolyl tetrazolium (MTT) assay.

### Cellular uptake and colocalization with p-tau

HT22 cells were seeded into 12-well plates at a density of 2 × 10^5^ cells per well overnight. After incubation with the various 5 μM COU 6-labelled formulations for 4 h at 37 °C, the cells were washed in PBS three times, fixed in 4.0% paraformaldehyde for 15 min at room temperature, and then incubated with 10 µg/mL Hoechst 33258 for 15 min. The fluorescent images of the cells were analyzed by confocal laser scanning microscopy (CLSM). Furthermore, flow cytometry was used to quantitatively evaluate the cellular uptake of RBMVECs by HT22 cells that were seeded into 12-well plates at a density of 5 × 10^6^ cells per well overnight. After incubation with the various 5 μM COU 6-labelled formulations for 4 h at 37 °C, the cells were collected, washed twice with PBS, and then immediately analyzed by flow cytometry (FCM) (BD FACSCalibur, USA).

To explore the co-localization of p-tau with RITC-labeled nanoparticles in HT22 cells, the cells were prepared and grouped as described in the protocol above. Then, 5 μM COU 6-labeled PCNPs, RPCNPs and T807-RPCNPs were added to each confocal dish with OA and incubated for 4 h. COU 6-labeled PCNPs, RPCNPs and T807-RPCNPs were also added to normal cells and incubated for 4 h. After incubation, the cells were fixed in 4% paraformaldehyde for 10 min and incubated for 15 min in 0.5%Triton-X in PBS solution; then, the cells were incubated for 1 h in a blocking solution (5% BSA in PBS), and finally, were incubated with anti-Tau AT8 (Ser202, Thr205) antibody (Invitrogen) at 37 °C for 2 h. After they were washed with PBS three times, the cells were incubated for 1 h with a fluorescence-conjugated secondary antibody (TRITC-conjugated anti-rabbit IgG secondary antibody made in goat, Abcam). The samples were again washed with PBS three times. Finally, the samples were incubated with Hoechst 33258 (10 μg/mL) for 15 min and then washed with PBS three times. The fluorescence signals were observed by CLSM.

The article "Neuron tau-targeting biomimetic nanoparticles for curcumin delivery to delay progression of Alzheimer’s disease" was retracted in 2023. Reasons: manipulated images; errors in the images; original data or images not available; unreliable data.

### Antiphagocytic ability of biomimetic nanoparticles

RAW264.7 cells (2 × 10^5^ cells per well) were seeded into a culture dish with DMEM at 37 °C and a 5% CO_2_ atmosphere. After 24 h, the cells were incubated with various 5 μM COU 6-labelled biomimetic nanoparticles for 4 h. After the incubation, the cells were collected and fixed in 4% paraformaldehyde, after which the cell nuclei were stained with Hoechst 33258 for 15 min. The fluorescence images of the cells were analyzed via CLSM (UltraVIEW Vox, PerkinElmer, USA).

### Pharmacokinetic studies

The pharmacokinetic profiles of various CUR-loaded biomimetic nanoparticles were measured in SD (male, 220 ± 10 g, n = 3) rats with a single dose of 5 mg**/**kg CUR by tail vein injection. Free CUR diluted in 25% Tween 80 was injected in the other group of rats for pharmacokinetic comparison. Blood (0.5 mL) was sampled from the retro-orbital sinus at different time points. The extraction of CUR was performed as described previously [36], with minor modifications. Briefly, 10 µL of the internal standard (I.S.) solution (felodipine, 300 ng/mL) was added to 100 µL of plasma sample. The sample mixture was deproteinized with 0.8 mL of ethyl acetate and vortex-mixed for approximately 5 min, after which the precipitate was removed by centrifugation at 14,000 rpm (revolutions per minute) for 5 min. Then, 800 µL of supernatant was transferred to another clean test tube and evaporated to dryness at 40 °C with a CentriVap Concentrator. The dry residue was reconstituted in 100 µL of the mobile phase, vortex-mixed, and centrifuged at 14,000 rpm for another 5 min. The sediment was then dissolved in 100 µL methanol.

The CUR concentration in rat plasma was measured using an Agilent high-performance liquid chromatographic (HPLC)–electrospray ionization–tandem mass spectrometry system (Pump G1312C, Autosampler 1367E, Degasser G1322A, G6460A triple-quad mass spectrometer, Agilent Technologies, Santa Clara, CA, USA). Felodipine was used as the internal standard. Chromatographic separation was performed on a reversed phase C8 analytical column (Agilent Zorbax Eclipse XDB C8, 2.1 × 100 mm, 3.5 μm, Agilent Technologies, Santa Clara, CA, USA) under isocratic conditions using methanol containing 5 mM ammonium formate at a flow rate of 0.3 mL/min.

The article "Neuron tau-targeting biomimetic nanoparticles for curcumin delivery to delay progression of Alzheimer’s disease" was retracted in 2023. Reasons: manipulated images; errors in the images; original data or images not available; unreliable data.

The triple-quadrupole mass spectrometer was operated in positive ionization mode, and detection and quantification were performed using multiple-reaction monitoring (MRM). MS/MS detection was conducted by monitoring the fragmentation of 369.1 → 177.0 (m/z) for CUR and 384.1 → 338.1 (m/z) for felodipine. The product ions were generated with collision energies of 20 eV and 5 eV for CUR and felodipine, respectively. Optimized MS parameters were as follows: fragment voltage, 140 V and 135 V for CUR and felodipine, respectively; capillary voltage, 4000 V; gas temperature, 300 °C; gas flow, 9 L/min; nebulizer pressure, 35 psi.

### Transport across BBB and targeting of nerve cells

The BBB model was established using Transwell plates [37], with minor modifications. Briefly, RBMVECs were plated on the apical side of the chamber at a density of 1.0 × 10^4^ cells per insert (Corning, NY, USA), and hen, As were seeded on the opposite side of the Transwell insert at a density of 1.0 × 10^4^ cells per insert. After incubation for 5 days (transendothelial electrical resistance, TEER exceeded 200 Ω/cm^2^), HT22 cells were seeded in the bottom of 12-well plates at a density of 1.0 × 10^3^/mL, and then 2 mL of DMEM containing OA (40 nM/L) was added to the bottom chamber (Additional file 1: Figure S4). Next, different 5 μM COU 6-tagged biomimetic nanoparticles were added to the apical compartment. After incubation for 6 h, fluorescent signals of the HT22 cells in the lower chamber were observed using CLSM and FCM.

### In vivo imaging

The near-infrared dye DIR was the fluorescent probe used to evaluate the brain-targeting efficiency of the nanoparticles in the OA-treated AD mice. Using a stereotaxic apparatus, the mice were injected with 1.5 µL OA (0.1 mg/mL) for 7 days after which they were administered various DIR-labelled biomimetic nanoparticle formulations by tail vein injection. Thirty minutes after the i.v. injection, in vivo imaging was performed with an IVIS^®^ Spectrum-CT. Fluorescent signals were quantified using Living Image^®^ software (Caliper, Alameda, CA).

### Western blotting

HT22 cells were pretreated with OA (40 nM) for 12 h and then treated with CUR-loaded PCNPs, RPCNPs, T807/RPCNPs, bare T807/RPCNPs or CUR for 12 h. The final concentration of each CUR was 5 μg/mL. The cells were then harvested and lysed with RIPA buffer (containing 1% protease inhibitor and 1% phosphatase inhibitor). Protein concentrations were determined using a BCA Protein Assay Kit. The proteins were separated by 10% SDS-PAGE and then transferred onto polyvinylidene difluoride membranes (PVDF, Millipore, USA). The membranes were incubated in 10% bovine serum albumin (BSA) for 1 h at RT and then incubated with the following primary antibodies for 3 h at RT: phosphor (p)-Tau (Ser 199, Thr 205, Ser 396), ERK 2, p-Gsk3β, p-Akt, β-Actin, Bax, and cleaved Caspase-3 (Abcam, USA). After the membranes were rinsed, they were incubated with the appropriate secondary antibodies for 1 h at RT, followed by detection using a Western Luminescent Detection Kit (Beijing Pulilay Gene Technology Co., Ltd. China). The sample bands were observed by enhanced chemiluminescence (ECL) detection reagents and analyzed by Quantity One; protein levels were normalized to the levels of β-actin and GAPDH.

The article "Neuron tau-targeting biomimetic nanoparticles for curcumin delivery to delay progression of Alzheimer’s disease" was retracted in 2023. Reasons: manipulated images; errors in the images; original data or images not available; unreliable data.

### Real-time quantitative RT-PCR analysis

HT22 cells were seeded onto T25 culture flasks (1 × 10^6^ cells/well) for 24 h. Then, 40 nM OA was added. After incubation for another 12 h, the medium was replaced with 5 mL of CUR-loaded PCNPs, RPCNPs, T807/RPCNPs, bare T807/RPCNPs or CUR overnight. The final concentration of each CUR was 5 μg/mL. The total RNA in the cells was collected using Trizol reagent (GIBCO BRL; Invitrogen, Carlsbad, CA) according to the manufacturer’s protocol. Then, the extracted RNA pellets were quantified, and first-strand cDNA synthesis was performed using a Fast Quant RT Kit (Tiangen biochemical technology co., Ltd, Beijing). Samples were tested by real-time PCR (Bio-Rad, USA) using a SYBR Green PCR master mix (Applied Biosystems, USA). The DNA product was amplified by primers and measured by real-time PCR. All primer sequences are presented in Additional file 1: Table S1.

### Total p-tau quantification in vitro and in vivo

HT22 cells were cultured in 12-well plates (1 × 10^6^ cells/well) before the medium was replaced with 2 mL of OA (40 nM/L). After incubation for 12 h, the cells were treated with free CUR, PCNP-CUR, RPCNP-CUR, T807/RPCNP-CUR, or T807/RPCNP, the final concentration of each CUR was 5 μg/mL. And then the cells were chipped and tested using a p-tau ELISA detection kit (Shanghai Heguo Biological Technology Co., Ltd. China). The AD mice were divided into six groups, after which they were intravenously injected with the different NPs described above with a CUR dosage of 5 mg/kg. Thirty minutes after i.v. injection, the mice were sacrificed, and all hippocampal tissues were separated and tested by a p-tau ELISA detection kit.

The article "Neuron tau-targeting biomimetic nanoparticles for curcumin delivery to delay progression of Alzheimer’s disease" was retracted in 2023. Reasons: manipulated images; errors in the images; original data or images not available; unreliable data.

### Mitochondrial ROS measurement

HT22 cells were cultured in 12-well plates (1 × 10^6^ cells/well) before the medium was replaced with 2 mL of OA (40 nM/L). After incubation for 12 h, the cells were treated with different CUR-loaded biomimetic NPs. The final concentration of CUR in each particle type was 5 μg/mL. The relative levels of mitochondrial ROS were measured using an ROS assay in which MitoSOX (Invitrogen Life Technologies, Carlsbad, CA) served as a fluorescent probe.

### Cell apoptosis assay

HT22 cells were seeded onto 6-well plates (1 × 10^6^ cells/well) for 24 h. Then, the medium was replaced with 2 mL of OA (40 nM**/**L). After incubation for 12 h, the cells were washed with PBS and exposed to fresh medium containing various CUR-loaded nanoparticles. Following 12 h of incubation, the cells were collected and stained using an Annexin V-FITC apoptosis detection kit (Beyotime Institute of Biotechnology, Jiangsu, China) according to the manufacturer’s instructions and were immediately analyzed by FCM.

### Morris water maze (MWM) behavioral test

The spatial memory function of the mice was tested by MWM. Mice in the experimental groups were slowly injected with 1.5 µL OA (0.1 mg/mL) using a stereotaxic apparatus [38], whereas mice in the control group were injected with 1.5 µL saline using the same apparatus. Seven days later, the experimental group was subjected to the MWM, which tested the memory impairment was screened in the mice. The mice were randomly divided into six groups (n = 20) and treated with 0.9% saline (control), free CUR or various biomimetic nanoparticle formulations carrying CUR by i.v. injection every other day for a total of 10 days at a CUR concentration of 2 mg**/**kg. The maze was composed of circular blue opaque plastic with a depth of 40 cm and a width of 120 cm and was filled with water, which was maintained at 25 °C ± 1 °C using an automatic heater to sustain a constant temperature. At the pool midpoint, two imaginary perpendicular lines crossed to divide the tank into four quadrants. A small platform (diameter 8 cm) was placed at a fixed position in the second quadrant 30 cm away from the perimeter and was hidden about 1.0 cm beneath the water surface. Some fixed visual cues were also placed around the wall of the maze. The performance of each mouse was recorded by a video-tracking system (JK001, Beijing Jinyuan Kechuang Technology Co., Ltd.), and data were calculated using software specific for the water maze. On the first 5 days, mice (n = 20 each group) performed three daily acquisition trials with a 20 min interval for 5 consecutive days. Briefly, three starting points, excluding the target quadrant, were randomly selected from three daily trials. Each mouse facing the wall of the tank was set free into the water. If a mouse failed to reach the platform within 60 s, it was then guided to the platform where it remained for a further 5 s. Within the intertrial interval, the mice were towel-dried. After three trials, the mice were removed from the water, towel-dried, and then returned to their home cage. The swimming speed, swimming path, and the escape latencies to find the platform were recorded. On the sixth day, the fixed platform was removed for a probe trial to test each mouse’s spatial memory. Each mouse was released into the water at the right opposite position of the target quadrant and permitted to swim freely for 60 s. Spatial acuity was determined according to the percentage of time spent in the target quadrant and the times required to cross the platform.

The article "Neuron tau-targeting biomimetic nanoparticles for curcumin delivery to delay progression of Alzheimer’s disease" was retracted in 2023. Reasons: manipulated images; errors in the images; original data or images not available; unreliable data.

### Concentration of CUR in the brain

The OA-treated mice were randomly divided into three groups (n = 7) and were intravenously injected with the following: free CUR, RPCNP-CUR, or T807/RPCNP-CUR at a CUR dosage of 5 mg/kg. Thirty minutes after i.v. injection, the mice were sacrificed, and their brains were removed and stored at − 20 °C before analysis. The amount of CUR in the brain was analyzed by LC–MS/MS, as previously described [39].

### Immunofluorescence staining

After the MWM test, six mice were randomly selected from every group and sacrificed, after which their brains were collected. The brains were fixed in 10% formalin and sectioned into 3 μm-thick slices. The brain tissue sections were incubated with the primary antibody in 5% BSA overnight at 4 °C, and staining was detected using TRITC-labeled secondary antibodies, as previously reported [40]. Finally, the images were captured via CLSM.

### Hematoxylin and eosin (H&E) staining

After we obtained immunofluorescence data, the remaining animals were sacrificed. A hematoxylin and eosin (HE) staining was performed according to previous reports [41]. Briefly, the mice were anesthetized with 10% chloral hydrate (350 mg/kg), i.p. Then the mice were perfused with 200 mL 0.9% NaCl solution and subsequently with 4% paraformaldehyde in 0.1 mol/L phosphate buffer at pH 7.4. Brains were removed and post-fixed for 24 h in the same fixative. The post-fixed brains were cryo-protected in 25% sucrose in PBS. Then the brains were removed, paraffin-embedded, and coronally sectioned at 8 μm thickness. The sections were then mounted on slides and stained with H&E. The cell loss of the hippocampal area was assessed and quantified under a microscope (Nikon eclipse E100, Japan).

### In vivo safety evaluation

Healthy mice were randomly divided into four groups (n = 6) and treated with 0.9% saline (control), free CUR, CUR-loaded RPCNPs or T807-RPCNPs by i.v. injection at a concentration of 2 mg/kg CUR. After 7 days, the mice were sacrificed, and samples of heart, liver, brain, spleen and kidney were collected and routinely stained with hematoxylin and eosin (H&E).

The article "Neuron tau-targeting biomimetic nanoparticles for curcumin delivery to delay progression of Alzheimer’s disease" was retracted in 2023. Reasons: manipulated images; errors in the images; original data or images not available; unreliable data.

### Statistical analysis

The data are presented as the mean ± standard deviation (SD). The difference between any two groups was determined using ANOVA. p < 0.05 was considered statistically significant.

## Results and discussion

### Synthesis and characterization of T807-RPCNPs

The RBCm (outer shell) was derived from RBC membranes and the NP (inner core) was prepared using a solvent displacement method. The resultant RBCm were coated onto the surface of NPs through mechanical extrusion to form RBCm-coated PLGA (RPCNP) NPs; these were then transferred to water after modification with amino-T807 (designated as T807/RPCNP-CUR NPs), which was obtained by conjugating amino-T807 to DSPE-PEG-NHS (Fig. 2a). The purified materials were obtained by dialysis (MWCO 3.5 kDa) against distilled water. Successful synthesis was evidenced by TOF–MS analysis (Fig. 2b). Transmission electron microscopy (TEM) revealed that the nanoparticles were successfully coated with RBCm and had a diameter less than 200 nm (Fig. 2d). After they were transferred to water, the hydrodynamic diameter and ζ-potential of each NP increased as they were coated with RBCm and modified with T807 and increased from 150 to 170 nm and from − 47.3 to + 8.9 mV, respectively. The observed size and surface potential changes confirmed the successful conjugation of T807 to the nanoparticles (Additional file 1: Table S2). The size and encapsulation are important factors for drug-loaded NPs to exert their functions. In this study, we prepared a high entrapment of CUR using an emulsion-solvent method. Compared with other techniques of PLGA nanoparticle production, such as salting-out, nanoprecipitation, and supercritical antisolvent precipitation, the emulsion-solvent evaporation method is the most frequently used method in the pharmaceutical industry to obtain a controlled release formulation [42]. The stability of T807/RPCNP-CUR NPs in physiological conditions is a precondition for their utilization in vivo. Therefore, PBS containing fetal bovine serum (FBS, 10% v/v) was used to simulate conditions in vivo. The stability of T807/RPCNP-CUR in PBS (containing 10% FBS) at 37 °C was estimated by the Turbiscan Lab Expert. According to the criteria of this instrument, the transmission and backscattering changes shown in Additional file 1: Figure S1 were less than 2%, which indicated that no distinct aggregations or sedimentations occurred in the release medium of T807/RPCNP-CUR after 24 h. This suggested that even though the T807/RPCNP-CUR NPs have a positive surface potential, their stability was not affected, which may be due to the steric stabilization of RBCm in the serum.

The article "Neuron tau-targeting biomimetic nanoparticles for curcumin delivery to delay progression of Alzheimer’s disease" was retracted in 2023. Reasons: manipulated images; errors in the images; original data or images not available; unreliable data.

**Fig. 2:** Preparation and characterization of nanoparticles. **a** Preparation of DSPE-PEG_3400_-T807. **b** MALDI-TOF mass spectra of DSPE-PEG_3400_-T807. Blue arrows represent the mass–charge ratios of DSPE-PEG_3400_-T807. **c** The release profiles of CUR, PCNP-CUR, RPCNP-CUR and T807/RPCNP-CUR in PBS (pH7.4, contain 10% FBS, v/v). **d** Morphological appearance of RBC, PCNP-CUR, RPCNP-CUR and T807/RPCNP-CUR based on TEM

The in vitro drug release profiles of CUR from the PCNP-CUR NPs and RPCNP-CUR NPs in PBS (pH 7.4, 37 °C) over 24 h are shown in Fig. 2c. Release profiles were obtained by presenting the percentage of drug released from these nanoparticles with respect to the amount of CUR encapsulated in the PLGA NPs. According to the curves, the release patterns of the T807/RPCNP-CUR NPs group is similar to those of the RPCNP-CUR NPs and PCNP-CUR NPs groups, in which drug release occurred in a biphasic manner, with an initial burst phase followed by a slower or sustained drug release phase compared with the free CUR group. The similarity in the drug release profiles of the three nanoparticles suggests that the T807 modification did not significantly affect the release profile of the CUR-loaded NPs.

### In vitro cell viability assay and cellular uptake

To assess the biosafety of these biomimetic NPs, we used a methyl thiazolyl tetrazolium (MTT) assay to investigate cytotoxicity of OA on HT22 cells. In this study, HT22 cells were used to evaluate the targeting effect of the constructed nanocarriers, as the cell lines have previously been used as neuronal-like cell models [43, 44]. We first screened the relative appropriate OA concentration using another MTT experiment and found that 40 nM OA could induce cell death, including apoptosis, in most HT22 cells. As illustrated in Fig. 3a, no obvious influence was found on the survival of HT22 cells after they were incubated with the different concentration of PCNPs, RPCNPs or T807/RPCNPs, which each contained different NPs but no OA for 12 h. The cell viability was above 90% in each group (Additional file 1: Figure S2), which demonstrated that the NPs were suitable for biological experiments. To ensure that we had enough cells for later experiments, the toxicity of different CUR-loaded NPs on OA-treated cells was investigated. When treated with OA, all these CUR-loaded NP groups showed higher cell viability than the OA group (Additional file 1: Figure S3). The cell viability in the RPCNP-CUR and T807/RPCNP-CUR groups were above 70%, 80% respectively, compared with the OA and the same concentration of free CUR groups. PCNP-CUR NPs exhibited lower cell viability than RPCNP-CUR and T807/RPCNP-CUR NPs (Fig. 3a), which indicated that the RBCm-coated NPs could enter neurons more readily than NPs without RBCm coating.

The article "Neuron tau-targeting biomimetic nanoparticles for curcumin delivery to delay progression of Alzheimer’s disease" was retracted in 2023. Reasons: manipulated images; errors in the images; original data or images not available; unreliable data.

**Fig. 3:** Cytotoxicity effect and specific tau targeting capability of biomimetic formulations. **a** The suitable concentration of OA for the model of AD after exposure to different concentration for 12 h, then the toxicity of different NPs on HT22 cells treated with or without 40 nM OA at a higher concentration. Error bars represent standard deviation. Statistical analysis was performed using a one-way ANOVA test, with *** indicating p < 0.001, ** indicating p < 0.01, and * indicating p < 0.05 (n = 6 per group). **b** The internalization of COU-tagged biomimetic NPs in HT22 cells (scale bar = 20 μm). **c** Confocal fluorescence images of different NPs in OA-treated HT22 cells after 4 h incubation. Cells stained with hoechst33258 are shown in blue fluorescence. The immunofluorescence staining of OA-treated HT22 cells with phosphor-tau AT8 (ser202, Thr205) antibody are shown in red fluorescence. COU-labeled PCNP, RPCNP and T807/RPCNP are shown in green fluorescence (scale bar = 50 μm)

Neurons are the targets of NPs modified with T807. The cellular uptake of T807-modified NPs and non-T807-modified NPs was evaluated by laser scanning confocal microscopy after incubation for 4 h. As shown in Fig. 3b, the fluorescence intensity of COU 6-labeled T807-modified NPs was remarkably higher than that of COU 6-labeled non-T807-modified NPs on HT22 cells, which implies that T807 significantly enhanced the cell uptake of NPs. This may be due to the high lipid content and positive surface potential of T807.

### p-tau-targeting

The p-Tau-targeting of T807/RPCNP-Cou 6 NPs in a neuronal-like cell model was monitored by confocal microscopy. HT22 cells were pretreated with OA for 12 h and then treated with different nanoparticles for another 4 h. Immunofluorescence staining with a p-tau antibody (AT8) demonstrated the up-regulation of tau phosphorylation in OA-treated cells. Figure 3c illustrates images of the co-localization of biomimetic nanoparticles with p-Tau in HT22 cells after treatment with various COU 6-tagged formulations. Firstly, we found that the cell uptake of T807/RPCNP-COU 6 by OA-treated HT22 cells was significantly higher than that of PCNP-COU 6 and RPCNP-COU 6 NPs, which indicates that this ligand could sufficiently improve its entry into the cells. This may be attributed to its positive surface charge, which allows for easy adherence to cell membrane surfaces. The fluorescence signal of COU 6-labeled T807/RPCNP overlapped with the immunofluorescence signal of AT8 (Ser202, Thr205) (Fig. 3c). Studies reported that T807 was bound to hyperphosphorylated tau with greater binding affinity [45]. Our data were in accordance with previous studies, which suggests that T807/RPCNP possesses the ability to target hyperphosphorylated tau in OA-treated HT22 cells and that using this target ligand for drug delivery is realizable.

The article "Neuron tau-targeting biomimetic nanoparticles for curcumin delivery to delay progression of Alzheimer’s disease" was retracted in 2023. Reasons: manipulated images; errors in the images; original data or images not available; unreliable data.

### The long circulation feature of biomimetic nanoparticles

Next, we performed sodium dodecyl sulfate (SDS)-polyacrylamide gel electrophoresis (PAGE) to examine the total protein components of these RBCm-coated NPs. The results showed that the compositions of membrane proteins were mostly preserved on RBCm-coated NPs during the modification process of the two ligands compared with empty RBCm-derived vesicles (Fig. 4a), including the integrin-related protein CD47 (Fig. 4b), which is a well-documented protein marker firmly embedded in the RBCm; this protein can inhibit macrophage phagocytosis through interaction with the SIRP-α receptor [46].

**Fig. 4:** The stealth properties of RBCm-coated NPs in vitro and in vivo. **a** SDS-PAGE of purified RBCm-coated NPs and emptied RBC membrane-derived vesicles (control). Samples were run at equal protein concentration and stained with Coomassie Blue. **b** CD spectra of RBC membranes, RPCNP and T807/RPCNP NPs. **c** CLSM images of RAW264.7 cells after incubation with various COU-tagged formulations. Scale bars represent 20 μm. **d** Plasma CUR concentration–time profiles after i.v. injection of different formulations in rat. The data are presented as the mean ± SD (n = 3)

Although most of the proteins were preserved on the surface of these NPs, whether they persisted in the blood despite the presence of macrophages still needs to be verified. To confirm whether T807/RPCNP NPs and RPCNP NPs inherit the long-term circulation feature of RBCm, an antiphagocytosis assay was performed in vitro. RAW264.7 murine macrophages were utilized as a cell model to determine the stealth capability of biomimetic NPs. After incubation with PCNP-CUR, RPCNP-CUR, or T807/RPCNP-CUR for 4 h, the fluorescence intensity of each cell group was determined by CLSM. From Fig. 4c, we see that the green signal in RAW264.7 cells treated with PCNP-CUR was extremely high compared with the RBCm-coated NPs and control treatment groups. The RPCNP-COU 6 and T807/RPCNP-CUR were not phagocytosed by RAW264.7 cells.

After the antiphagocytosis ability of the two biomimetic NPs was evaluated in vitro, the pharmacokinetics studies were conducted in vivo. HPLC–MS was used to monitor the concentration of CUR release in the blood. It was found that the level of plasma CUR in the free CUR group decreased sharply and could hardly be detected after 4 h. Without RBCm, the free CUR and PCNP NPs groups were rapidly eliminated from the bloodstream before they released sufficient CUR, which is vital to their treatment effect. In contrast, the plasma CUR level in biomimetic NPs (PCNP-CUR, RPCNP, T807/RPCNP) decreased slowly within 12 h compared with the free CUR group (Fig. 4d). As shown in Additional file 1: Table S4, CUR-loaded biomimetic formulations (RPCNP, T807-RPCNP) displayed curves resembling pharmacokinetic curves, and no significant difference was observed in the T_max_, C_max_, t_1/2_, MRT, CL and AUC_(0−t)_ between these formulations (p > 0.05). Compared with PCNP-CUR, the spectacular increase in T_max_, C_max_, t_1/2_, MRT, and AUC_(0−t)_ and the decrease in CL were also visible. All these results demonstrated that RBCm-coated NPs were associated with a significantly prolonged circulation of CUR in blood. Simultaneously, modification with the T807 ligand did not affect the long-term circulation of the biomimetic NPs. The in vitro and in vivo experiments indicated that the preparation method of the RBCm did not destroy the structure of important surface proteins.

The article "Neuron tau-targeting biomimetic nanoparticles for curcumin delivery to delay progression of Alzheimer’s disease" was retracted in 2023. Reasons: manipulated images; errors in the images; original data or images not available; unreliable data.

### Transport across the BBB

Good in vitro blood–brain barrier (BBB) permeation is essential for brain targeting delivery systems. The transport capacity of different NPs across the BBB was evaluated by Transwell experiments in vitro and by live imaging in vivo. RBMVECs, As and HT22 cells were used to mimic the BBB in vitro, and when As and RBMVECs were co-cultured, the TEER reached 261.2 ± 3.1 Ω/cm^2^ (Additional file 1: Table S3). After HT22 cells were added, the TEER reached 381.9 ± 6.2 Ω/cm^2^ (exceeded 200 Ω/cm^2^), which signified that the three co-cultured cell lines demonstrated good barrier function for evaluating the transport of these NPs across the BBB. From Fig. 5a, b, we found that small amounts of fluorescence signal were acquired after treatment with Control, PCNP-COU 6 or RPCNP-COU 6. In contrast, the fluorescence signal from T807/RPCNP-COU 6 was markedly evident at the same time, which shows that T807/RPCNP-COU 6 has the ability to cross the BBB. The results demonstrated that the increased permeation of the BBB to RPCNP in an in vitro COU 6 model was attributed to the T807 modification, which suggests that T807/RPCNP NPs could be a suitable drug delivery system for AD treatment.

**Fig. 5:** Transport across the BBB of biomimetic formulations in vitro and in vivo. **a** CLSM images of HT22 cells after incubation with different COU-tagged various formulations acrossing As and RBMVEC two co-culture cells, which contain COU (green) and Hoechst 33258 (Blue, nuclear imaging). **b** FCM quantification of various COU-tagged (Green) formulations in HT22 cells. **c** In vivo brain-targeting ability. Biodistribution of DIR contained in various formulations in AD model mice determined by an IVIS^®^ Spectrum. **d** The mice were sacrified and the fluorescence in various organs was detected

Along with in vitro BBB permeation, NPs that crossed the BBB in vivo to target the brain were evaluated by live images. From Fig. 5c, d we learned that after OA treatment, only the mice injected with DIR-tagged T807/RPCNP NPs exhibited a significant fluorescence signal in the brain compared with the other NPs, and moreover, the fluorescence signal in brain tissues was the same as that in the 3D live images. The above experimental results strongly indicated that the T807-modified NPs could be effectively transported across the BBB and aggregated in neuronal p-tau site.

The article "Neuron tau-targeting biomimetic nanoparticles for curcumin delivery to delay progression of Alzheimer’s disease" was retracted in 2023. Reasons: manipulated images; errors in the images; original data or images not available; unreliable data.

### Inhibition of tau hyperphosphorylation and aggregation

One of the primary components of AD-associated NFTs is aggregated tau [47]. Aggregated tau has been discovered to be hyperphosphorylated, and thus reducing the phosphorylation level of tau is very important for delaying the pathogenesis of AD [48]. Restraining tau aggregation is also vital to AD treatment. The total p-tau level in HT22 cells was tested by ELISA, as shown in Fig. 6a, the OA-treated HT22 cells exhibited a high level of p-tau compared with the control group, but after treatment with CUR-loaded NPs, the level of p-tau was greatly decreased. Most of all, the T807/RPCNP-CUR group showed the most obvious trend in decreasing p-tau level, which means that T807/RPCNP-CUR exerted the best effect on tau aggregation and the resulting trends coincided with the CLM results.

**Fig. 6:** Therapeutic effect of CUR-loaded biomimetic formulations in vitro. **a** p-tau Elisa kit analysis of cellular total p-tau level after treated with different formulations in OA-treated HT22 cells. **b** Western blot and **c** quantification results for hyperphosphorylated tau at threonine 205 epitopes, serine 396 and 404 epitopes in HT22 cells. Statistical analysis was performed using a one-way ANOVA test, with *** indicating p < 0.001, ** indicating p < 0.01 and *indicating p < 0.05 compared to the OA group (n = 3 per group). Error bars represent standard deviation

In AD, the pattern of phosphorylation changes as the disease progresses, and thus we performed a western blot to monitor the p-tau level at multiple sites (serine 396, 404, and threonine 205) in OA-treated HT22 cells to test whether our NPs loaded with CUR could down-regulate the hyperphosphorylated tau level (Fig. 6b) [49]. As CUR prevented tau aggregation and reduced the p-tau level [50], the WB results also indicated that the groups containing CUR significantly reduced the p-tau level in OA- treated cells (Fig. 6c). However, the T807/RPCNP-CUR had a better effect on the downregulation of the p-tau level than the two other groups, as seen in Fig. 6b, c. Concurrently, we also found that compared with the OA-treated group, the T807/RPCNP NPs without CUR had no effect on these hyperphosphorylation sites, especially S396, the phosphorylation of which is one of the earliest events in AD, which suggests that our T807-modified empty carrier did not participate in the depression of the hyperphosphorylated tau level.

The article "Neuron tau-targeting biomimetic nanoparticles for curcumin delivery to delay progression of Alzheimer’s disease" was retracted in 2023. Reasons: manipulated images; errors in the images; original data or images not available; unreliable data.

### Relieving OA-induced oxidative stress

Hyperphosphorylated tau induces tau aggregation in AD; tau aggregation in turns leads to the formation of NFTs, which aggravates the pathogenesis of AD and neuronal mitochondrial damage. The release of ROS by damaged mitochondria aggravates tau pathology and the AD process [51]. From the FCM results (Fig. 7a), we can see that our T807/RPCNP-CUR could significantly inhibit mitochondrial ROS (mitoROS) release in OA-treated HT22 cells compared with the other groups. The confocal images further confirmed the outstanding ROS scavenging ability of T807/RPCNP-CUR.

**Fig. 7:** Cytoprotection effect of biomimetic formulations in vitro. **a** FCM analysis of mitochondrial ROS accumulation in HT22 cells obtained by MitoSOX. **b** Apoptosis results of HT22 cells after treatment with different CUR-loaded formulations. Cells were stained with Annexin V-FITC/PI

### Protecting neurons from apoptosis

Apoptosis is known to play a crucial role in neuronal loss in AD and in the induction of ROS release; therefore, the increased tau aggregation significantly implicates induction of an apoptotic response [52]. Therefore, in our study, we examined the antiapoptotic ability of T807/RPCNP-CUR by FCM, and used free CUR and RPCNP-CUR as the contrast groups in OA-treated HT22 cells (Fig. 7b). After OA treatment, the number of apoptotic cells (37.5%) was 2.5-fold higher than that of the control (15.0%), means that OA has a significant effect of inducing the apoptosis of neuronal-like cells. We also found that the free CUR and RPCNP-CUR groups had a similar antiapoptotic effect. Furthermore, T807/RPCNP-CUR exhibited the best antiapoptotic effect with a higher cell survival (73.7%) rate and a lower apoptosis rate (15.0%). The benefits of T807/RPCNP-CUR in the protection of neuronal-like cells from apoptosis may be ascribed to its ability to down-regulate hyperphosphorylated tau level and mitoROS release (The raw data are seen in Additional file 2).

The article "Neuron tau-targeting biomimetic nanoparticles for curcumin delivery to delay progression of Alzheimer’s disease" was retracted in 2023. Reasons: manipulated images; errors in the images; original data or images not available; unreliable data.

### Activation of PKB/GSK-3β signaling and regulation of apoptosis-relevant proteins

The above results confirmed that CUR-loaded T807/RPCNP could decrease the p-tau level, inhibit ROS release and restrain apoptosis of OA-treated neuronal-like cells. To further explore the underlying mechanism of CUR-loaded T807/RPCNP to protect cells against AD, we performed WB and RT-PCR to detect expression at the cellular level. Glycogen synthase kinase-3 (GSK-3) is a pivotal molecule in the progression of AD and is involved in the formation of paired helical filament (PHF)-Tau [53]. Phosphorylated protein kinase B (PKB) is also an important kinase in AD tau pathology. In addition, PKB is an upstream kinase of GSK3β, and thus PKB activation could restrain GSK3β expression and delay the progression of tau pathology. Since okadaic acid (OA) is a potent and selective inhibitor of the protein phosphatases PP1 and PP2A, it can induce hyperphosphorylation of tau and cause AD-like pathology [54]. Our results also confirmed that after OA treatment, p-PKB was reduced and GSK3β was increased in HT22 cells, but the opposite was observed in the free CUR and CUR-loaded RPCNP groups (Fig. 8a, b), which implies that CUR can regulate the PKB/GSK3β pathway. To investigate whether the T807 ligand modification of biomimetic nano-carriers participates in the mechanism of CUR in the treatment of AD, we used bare T807/RPCNP as the control group. Western blot results showed that CUR-loaded T807/RPCNP significantly upregulated PKB protein and downregulated GSK3β protein, but the bare T807/RPCNP did not have any effect on these two proteins, which suggests that bare T807/RPCNP did not affect the PKB/GSK3β pathway (Fig. 8a, b). We also found that the CUR-loaded T807/RPCNP treatment group had a better effect on the regulation of PKB and GSK3β than the CUR treatment group, which may be due to the nano-carrier’s slow release profile.

**Fig. 8:** In vitro therapeutic mechanism of biomimetic formulations in an OA-induced cell model. **a** Western blot and quantification results of Bax, Caspase 3, p-ERK 2 p-PKB, GSK3β, in HT22 cells after treatment different formulations. **b** Relative intensity of Bax, Caspase 3, p-ERK 2 p-PKB, GSK3β in HT22 cells with WB results. **c** Relative ratio of gene expression of *bax, caspase 3, erk, pkb, gsk3β* in HT22 cells after treatment with different formulations. Statistical analysis was performed using a one-way ANOVA test, with *** indicating p < 0.001, ** indicating p < 0.01 and *indicating p < 0.05 compared to the OA group (n = 3 per group). Error bars represent standard deviation

Over-expression of active ERK2 has been shown to reduce neuronal apoptosis in AD via modulating the expression levels of Bax and Caspase 3 [55]; we therefore explored the possibility that T807/RPCNP-CUR reduced apoptosis in an AD model, and we also explored the mechanism. In line with previous reports, the expression of both Bax and Caspase 3 was significantly decreased in the CUR and CUR-loaded NP treatment groups (Fig. 8a, b), especially in the T807/RPCNP-CUR group. WB results demonstrated that OA stimulated an increase in apoptosis-related proteins, which was reversed by T807/RPCNP-CUR; this suggests that T807/RPCNP-CUR provides protection against the initiation of apoptosis. The mRNA levels of PKB, GSK3β, Bax, and Caspase 3 were further confirmed by RT-PCR (Fig. 8c). Overall, T807/RPCNP-CUR rescued neuronal-like cells from apoptosis by activating the Akt/GSK3β pathway, inhibiting tau hyperphosphorylation and restraining ROS release. Moreover, pro-apoptotic proteins and related genes were also regulated by ERK2 activation.

The article "Neuron tau-targeting biomimetic nanoparticles for curcumin delivery to delay progression of Alzheimer’s disease" was retracted in 2023. Reasons: manipulated images; errors in the images; original data or images not available; unreliable data.

### In vivo therapeutic effect

With advantages in suitable physiochemical properties, long-term circulation, p-tau-targeting abilities, safety in vitro, and antiapoptotic effects, we subsequently evaluated the effect of CUR-loaded T807/RPCNP NPs in alleviating the progression of AD pathology. The MWM test was used to assess whether the CUR-loaded biomimetic nanoparticles could improve spatial learning ability in AD mice. The mean velocity of the mice in each group was not different (Fig. 9a). We also found that after injection with 2.5 µL OA (0.2 µg/µL) for 7 days, the mice exhibited impaired spatial learning and memory, as indicated by increased escape latency in finding the hidden platform in the navigation test and reduced retention time in the target quadrant in the probe trial test compared with the control mice (Fig. 9b–d). Encouragingly, after injection with T807/RPCNP-CUR, the mice exhibited improved spatial learning and memory in the two tests (Fig. 9b–d), and furthermore, the retention time and times to cross the platform in the target quadrant were also increased (Fig. 9c, d). The swimming path tracings of mice in different groups also affirmed that T807/RPNPC-CUR could accumulate in the brain. These positive results are due to the good permeability of the BBB to T807. After the mice were tested in the MWM, their brain tissues were extracted, and we detected the total p-tau level in the hippocampal region using a p-tau ELISA kit. Additional file 1: Figure S5 indicates that after injection of OA into the hippocampal CA1 region, the total p-tau in hippocampal tissue had increased approximately 4.1-fold that of the control. However, when mice were intravenously injected with T807/RPCNP-CUR, the total p-tau level was significantly reduced, and the same positive results verified that our CUR-loaded T807-modified nanoparticles could cross the BBB and improve cognitive impairment in AD mice.

The article "Neuron tau-targeting biomimetic nanoparticles for curcumin delivery to delay progression of Alzheimer’s disease" was retracted in 2023. Reasons: manipulated images; errors in the images; original data or images not available; unreliable data.

**Fig. 9:** In vivo therapeutic evaluation of CUR-loaded biomimetic formulations 1. **a** Mean velocity of mice in different formulation groups. **b** Escape latency time of each group. **c** The frequency of platform crossing at the final day with the platform removed. **d** Relative time spent on the target quadrant. **e** Representative swimming path tracings of mice in different groups. The data are presented as the mean ± SD (n = 20). * indicates p < 0.05, ** indicates p < 0.01, *** indicating p < 0.001

We then verified neuronal cell death by H&E staining and found that T807/RPCNP-CUR treatment significantly reduced neuronal cell death in the hippocampal CA1 region compared with the OA group, as seen in Fig. 10.

**Fig. 10:** Identification of neuronal survival in the hippocampal CA1 region after i.v. injection of with different CUR-loaded formulations in AD model mice. The data are presented as the mean ± SD (n = 5). ** indicates p < 0.01. *** indicates p < 0.001

Astrocyte and microglia are the principle nerve cells in the brain, and their activation is a key component of the cellular response to neurodegenerative disease, including AD [56]. Glial fibrillary acidic protein (GFAP) is expressed in astrocytes and ionized calcium binding adapter molecule-1 (Iba-1) is expressed in microglia. Upregulation of GFAP and Iba-1 is considered a surrogate marker of neuronal stress and inflammatory response in the brain. Downregulation of GFAP and Iba-1 protein expression and then elimination of microglia and astrocytic activation might be therapeutically beneficial in AD. Therefore, we further analyzed the effect of CUR-loaded T807/RPCNP on inflammation related to astrocytic and microglial activation in mice after the MWM test. Even though glial activation may exhibit anti-inflammatory properties against harmful stimuli [57], the swimming performance of mice in OA group showed that the abnormal activation of microglia aggravated the impairment of cognitive function. And as shown in Fig. 11, T807/RPCNP-CUR significantly inhibited abnormal activation of microglia and astrocytes compared with other formulations. These results suggested that CUR-loaded T807/RPCNP could mitigate brain inflammation by downregulating the p-tau level and ROS release.

**Fig. 11:** Immunohistochemical staining with GFAP, Iba-1 in each group, quantification of GFAP and Iba-1 positive cells in the corresponding images. Scale bars represent 100 μm. The data are presented as the mean ± SD (n = 5). * indicates p < 0.05. ** indicates p < 0.01

The article "Neuron tau-targeting biomimetic nanoparticles for curcumin delivery to delay progression of Alzheimer’s disease" was retracted in 2023. Reasons: manipulated images; errors in the images; original data or images not available; unreliable data.

### T807/RPCNP NPs increased CUR accumulation in the brain

It is known that CUR has poor bioavailability in vivo, especially in the brain. After the MWM, we conducted an experiment to test the concentration of CUR in the brain by HPLC–MS, and as shown in Additional file 1: Figure S6, we found that the CUR concentration in the brain was 6.3-fold higher than that of free CUR after injection with T807/RPCNP-CUR biomimetic NPs, which indicates that T807 had a strong brain- targeting ability. We can also see that even though CUR-loaded RPCNP increased the delivery efficiency of CUR in the brain compared with free CUR, the concentration of CUR in the brain was still unsatisfactory without T807. This result once again suggested that T807 is a potential clinically relevant target ligand that can be used to deliver CUR to the brain.

### In vivo safety evaluation

A good nano-carrier should have good biocompatibility and low toxicity in vivo. Here, we investigated the systemic toxicity of CUR-loaded T807/RPCNP, RPCNP, and free CUR in healthy mice with a high dose (20 mg/kg, every 2 days, by intravenous injection) (Fig. 6d). No significant differences in body weight were found between the NP-treated groups and the saline groups (Additional file 1: Figure S7). To further verify the toxicity of different NPs on the major organs of mice, the heart, liver, spleen, lungs, kidneys and brain were harvested and stained with hematoxylin and eosin (H&E). As is shown in Fig. 12, no obvious pathological features were seen in any of the organ systems in the NP-treated group and the two other contrast groups, which suggests that free CUR, CUR-loaded RPCNP and CUR-loaded T807/RPCNP did not cause systemic toxicity after i.v. injection with the current dosage. Moreover, we found similar results in the above experiments between the RPCNP and T807/RPCNP groups, which indicates that T807 did not significantly affect the biocompatibility of these biomimetic nanoparticles. Overall, these tests confirmed that T807/RPCNP has low toxicity and good biocompatibility in vivo, which is possibly due to the biodegradation of the “inner core” and the endogenous properties of the “outer shell”.

**Fig. 12:** Histological staining of organs from healthy mice treated with different CUR-loaded formulations

## Conclusions

In this study, we synthesized relatively small, positively charged T807/RPCNP NPs capable of crossing the BBB and localizing to p-tau in neurons. CUR-loaded T807/RPCNP NPs are biocompatible and can decrease the intracellular p-tau level, suppress neuronal-like cells death and scavenge ROS efficiently to alleviate AD progression in vitro and in vivo. The nano-carrier T807/RPCNP does not alter the anti-AD mechanism of CUR. Our results demonstrate a novel target strategy for the development of tau-targeting therapeutics against tau pathology and have important implications for the treatment of AD and other neurodegenerative diseases. This targeting strategy may be able to be used clinically by effectively delivering CUR to the brain. Although preliminary, the results of this work suggest that T807/RPCNP NPs might provide a potential intravenous neuronal tau-targeting delivery platform for the treatment of AD, there is lack of sufficient data in the experiment of CUR accumulation in the brain. In a future study, we will perform in vitro and in vivo studies to examine the p-tau targeted delivery mechanism and further conducting more proper experiments on targeting brain.

The article "Neuron tau-targeting biomimetic nanoparticles for curcumin delivery to delay progression of Alzheimer’s disease" was retracted in 2023. Reasons: manipulated images; errors in the images; original data or images not available; unreliable data.

## Supplementary information

**Additional file 1: Table S1.** Real Time PCR Primers and Conditions. **Table S2.** Characteristics of the biomimetic nanoparticles (NPs). **Table S3.** Pharmacokinetic parameters of different biomimetic NPs. **Table S4.** Transendothelial electrical resistance of co-culture cells. **Figure S1.** Stability of various biomimetic formulations in the presence of 10 % FBS in PBS at 37 °C. The delta transmission (∆T) and backscattering (∆BS) profiles were measured at each time point using a Turbiscan Lab^®^ Expert analyser. **Figure S2.** Cytotoxicity of PCNP(a), RPCNP (b), T807/RPCNP (c) NPs at different concentrations in HT22 cells. **Figure S3.** Inhibition of OA-induced cell death of HT22 cells after exposure to 40 nM OA for 12 h and then treated with different concentration of CUR(a), PCNP-CUR(b), RPCNP-CUR(c), T807/RPCNP-CUR(d) and T807/RPCNP(e) for another 12 h. **Figure S4.** An in vitro blood–brain barrier (BBB) model being composed of co-culture with endothelial (RBMVEC), astrocyte (As) and HT22 cells was established to evaluate the transcytosis of biomimetic formulations. **Figure S5.** Total p-Tau levels after treatment by different CUR-tagged formulations in OA-induced AD mice. The data are presented as the means ± SD (n = 5). ** indicates p < 0.01, *** indicates p < 0.001. **Figure S6.** The distribution of CUR in brain 0.5 h after i.v. injection. The data are presented as the means ± SD (n = 7). * indicates p < 0.05. ** indicates p < 0.01. **Figure S7.** Body weight in healthy mice after treatments with various CUR-loaded formulations. The data are presented as the means ± SD (n = 6).

**Additional file 2.** Raw data of mitoROS and apoptosis that measured by flow of cytometry.
